The article "Smart Garden Planning and Design Based on the Agricultural Internet of Things" was published in 2022. Journal: Comput Intell Neurosci.

# Smart Garden Planning and Design Based on the Agricultural Internet of Things

**DOI:** 10.1155/2022/8522751

**Published:** 2022-01-07

**Authors:** Yi Xun, Guangpei Ren

**Affiliations:** School of Art and Design, Guangdong University of Technology, Guangzhou, Guangdong 510060, China

## Abstract

To improve the effect of urban agricultural garden landscape planning and design, this paper combines the agricultural Internet of Things technology to construct a smart garden planning and design system. Moreover, this paper selects the LEACH protocol that can support monitoring for a long time according to actual application needs, introduces the latest swarm intelligence optimization algorithm, the gray wolf algorithm, to optimize some of the problems in the LEACH protocol, and conducts simulation experiments on the improved algorithm. The simulation experiment results show that the improved algorithm has obvious advantages in cluster head selection, data transmission within the cluster, and route maintenance. After constructing a smart garden planning system based on the agricultural Internet of Things, the effect of the agricultural Internet of Things data processing in this paper is evaluated. Finally, this paper constructs a garden simulation system and analyzes the performance of the system. The results verify that the agricultural Internet of Things has a good effect in the planning and design of smart gardens.

## 1. Introduction

Ecological culture is a new cultural outlook that represents new trends and trends in the world. It represents the awakening of human beings from the ignorant concept of ruling and conquering nature, seeking a way to respect and coexist in harmony with nature. It is the “ecological” and “natural” transformation of the central values of mankind [1].

Regarding the definition of the term landscape, many scholars have put forward different interpretations. In the field of landscape ecology, it studies the ecosystem of the entire natural world, and it focuses on the interaction between ecological subsystems such as climate, geology, soil, vegetation, hydrology, animal and human activities, and their impact on nature. In addition to studying the characteristics of the objective laws of the generation, development, and evolution of the landscape ecosystem itself, it also seeks measures and ways to rationally utilize, protect, and manage the landscape. The field of landscape geography focuses on the changes of natural landscape morphology, emphasizes the natural characteristics of the landscape, and pays attention to the development and evolution of landscape morphology and landform. From the perspective of landscape architecture, it focuses on the relationship between humanity and nature from the relationship between human and landscape and social attributes. The connotation of the landscape shows obvious characteristics of dynamic changes with the influence of human activities and the change of regional form. From the perspective of the entire development history of human society, the landscape on the Earth is the result of human adaptation and transformation of the natural world [2]. From the definitions of the three major disciplines mentioned above, it can be summarized that landscape is the trace left on the land by human activities or the interaction between humans and nature. The landscape can be regarded as an organic collection composed of a series of symbolic landscape elements. The landscape elements are the unit elements that make up this large collection of landscapes. Therefore, landscape elements can be divided into two categories: natural landscape elements and artificial landscape elements. Natural landscape elements include terrain, soil, vegetation, and Fengshui patterns, and artificial landscape elements include road paving, sketches, and buildings [3].

The article "Smart Garden Planning and Design Based on the Agricultural Internet of Things" was published in 2022. Journal: Comput Intell Neurosci.

In recent years, rural revitalization has been a key work and policy measure in my country. Rural complexes are an important measure to realize rural revitalization. Since the concept of rural complexes was put forward, many cities and towns in my country have been put into practice. However, research on rural complexes and the development of on-site projects is not perfect, and the aspects involved are relatively limited, mainly including leisure and entertainment, physiotherapy, sightseeing agricultural picking, and specialty catering. There are relatively few research studies and analyses on building a smart pastoral complex from the perspective of global tourism combined with the Internet of Things. Global tourism is not the same as previous tourism, blindly pursuing the growth of tourist visits, but focusing more on the improvement of tourism quality. Above all, global tourism aims to build tourism into tourism that can improve people's quality of life and also pursue the value of tourism in people's new wealth revolution.

Taking the agricultural pastoral as the theme, this paper combines the agricultural Internet of Things technology to carry out smart garden planning and design, so as to promote the development of the industry and raise people's awareness of ecological protection and bring people a good pastoral scenery experience.

## 2. Related Work

With the continuous development of spatial geographic information acquisition technology and computer communication technology, the amount of geographic information data continues to expand, and the difficulty of information extraction and analysis continues to increase. Geographic information has gradually changed from a “digital city” to a “smart city” [4]. At present, various countries are developing smart city projects in line with their own national conditions, such as smart grids in the United States and smart communities in the European Union. With the gradual maturity of 3D geographic information technology, 3D geographic information data have finally entered a wide range of applications in recent years, new stage [5]. In terms of data acquisition methods, noncontact rapid batch acquisition of large-scale data has been achieved at home and abroad. Oblique photography technology, which uses multisensor or dynamic sensors to synchronously collect images from the air, can collect rich high-resolution texture data on the surface and side of buildings and is an upgrade to the traditional single-sensor acquisition method of aerial photography [6]. Literature [7] shows a 3D map made with oblique photography data. At present, the AOS system in the United States, the Penta-DigiCam system in Germany, the A3 system in Israel, and the RCD30 in Leica in Germany are widely used internationally [8].

The article "Smart Garden Planning and Design Based on the Agricultural Internet of Things" was published in 2022. Journal: Comput Intell Neurosci.

With the popularization of drone technology, tilt photography technology has also shown explosive growth [9]. Now, in the smart city 3D modeling project, the oblique photography 3D modeling program has taken a place [10]. In addition, LiDAR technology, namely, laser scanning, has also emerged in many fields. It can quickly obtain high-precision point cloud data and is widely used in many fields such as surveying and mapping, architecture, deformation monitoring, mechanical engineering, archaeology, cultural relics protection, and autonomous driving [11]. At present, common international laser scanners include German ATOS 3D optical scanner, Swiss Leica 3D laser scanner, Austria RIEGL laser measurement system, and American Trimble 3D laser scanner [12].

In recent years, high-resolution satellite remote sensing technologies have also been continuously developed, such as QuickBird and WorldView in the United States. In my country, the Chinese “High Score Family” represented by Gaofen No. 2, No. 3, and No. 4 also provides reliable DOM (Digital Orthophoto) and DEM (Digital Elevation Model) for smart city 3D modeling projects data [13]. In the use of oblique photography data for 3D automatic modeling, there are foreign Smart3DCapture, Pixel Factory, PhotoMesh, PohtoScan, etc., which are all powerful tools suitable for the rapid production of smart city 3D models [14]. In the use of laser point cloud data for 3D automatic modeling, the current use of refined reverse engineering modeling software is mainly not suitable for the automatic production of large-area smart city 3D model data [15].

The article "Smart Garden Planning and Design Based on the Agricultural Internet of Things" was published in 2022. Journal: Comput Intell Neurosci.

The massive data of smart cities need to be supported by software platforms with spatial management and analysis functions, such as SkylineGlobe, ArcGlobe, CityEngine, etc., which are all currently used smart city geographic information platforms [16].

Smart city 3D models have a wide range of data sources, different production methods, and data structures. Only when a unified standard specification is formulated, can the data interoperability be realized [17]. The Open Geospatial Consortium (OGC) has established the 13S standard as a new international three-dimensional standard, which is a standard specifically designed for three-dimensional spatial geographic information data [18].

## 3. Agricultural Wireless Sensor Network Model

In order to make the research on wireless sensor networks more targeted, the research content in this article is based on the following assumptions:

- The sink node is located in the monitoring area, and its energy is continuously supplied by an external power source. It has stronger computing and storage capabilities than ordinary nodes, can connect to the external network, send data to remote observers, and maintain communication with at least one node in the network.
- The scale of the sensor network is designed to be 200 nodes, and they are randomly and evenly distributed in the monitored area. The nodes have limited energy and are supplied by their own batteries. They have certain computing and storage capabilities, and can sense their own remaining energy, and follow the network operation. As time progresses, the energy consumption of each node is not the same, and the energy of the nodes will be inconsistent.
- After the node is deployed, once the network is started, the position of the node will no longer change, and the node can know the distance between itself and other nodes through RSSI.
- All nodes have similar communication capabilities and data processing capabilities, there is no super node, the channels between the nodes are symmetrical, the node's transmission power is limited, and it has a unique ID code.
- The communication success rate of all nodes conforms to formula (1). There is a communication path with a hop count of *h* in the network. If it is assumed that the communication distance of the i-th hop is *d* and the effective communication distance of the node is *r*, then the communication success rate obeys the following formula [19]:

(1) $$\begin{array}{c} P_{\text{suc}}\left(h\right)=\prod_{i=1}^{h}p\left(d_{i}\right)=\frac{{\left(0.2\right)}^{h}d^{h},d^{h},\ldots ,d^{h}}{r^{h}}\leq 0.2^{h}. \end{array}$$

It can be seen from formula (1) that the fewer the number of hops, the shorter the path and the higher the communication success rate [20].

The article "Smart Garden Planning and Design Based on the Agricultural Internet of Things" was published in 2022. Journal: Comput Intell Neurosci.

The wireless sensor network communication channel is a random channel.

(2) $$\begin{array}{c} E_{\text{Tx}}\left(k\;d\right)=E_{\text{elec}}\left(k\right)+E_{mp}\left(k\;d\right)=\left\{\begin{array}{c} kE_{\text{elec}}+k\varepsilon d^{2},\;d\leq d_{0},\\ kE_{\text{elec}}+k\varepsilon d^{4},\;d\geq d_{0}. \end{array}\right. \end{array}$$

Here, *E*_elec_ is the receiving module to complete a complete transceiver, *ε*_*fs*_ and *ε*_*mp*_ depend on the parameters of the transmitting circuit and the receiving circuit, *d* is the distance between the transmitting node and the receiving node, and the calculation formula of *d*_0_ is as follows:

(3) $$\begin{array}{c} d_{0}=\sqrt{\frac{\varepsilon_{fs}}{\varepsilon_{mp}}}. \end{array}$$

*d*_0_ is the distance threshold. When *d* is less than *d*_0_, the communication of the node obeys the free space model.

(4) $$\begin{array}{c} E_{rx}\left(k\right)=kE_{\text{elec}}. \end{array}$$

The LEACH protocol is a WSN hierarchical routing protocol, which occupies a very important position in the research of WSN routing protocol.  Figure 1 is a schematic diagram of LEACH protocol clustering. Clustering algorithms such as DCHS, TEEN, and APPTEEN, all borrow the idea of LEACH algorithm. The LEACH algorithm first puts forward the idea of “round.” Each round is divided into two stages: cluster establishment and data transmission.

During the formation of the cluster, if the node randomly chooses a number between 0 and 1 and if the selected number is less than the threshold *T*(*n*), it is selected as the cluster head. The calculation formula of *T*(*n*) is as follows [21]:

(5) $$\begin{array}{c} T\left(n\right)=\left\{\begin{array}{cc} \frac{x}{l-x\left(r\mathrm{mod}\left(l/x\right)\right)}, & \mathrm{if}\;n\in S,\\ 0, & \text{otherwise}. \end{array}\right. \end{array}$$

At this point, one cycle is over and preparations for the next cycle are started.

Figure 2 is the LEACH protocol flowchart. First, the algorithm selects the cluster head node. After this cluster head is determined, a broadcast message is sent to other nodes. The message includes the cluster head location, cluster head ID, and energy information. The noncluster head node selects the cluster head closest to its position to join according to the received message to form a cluster, and the cluster establishment phase is completed. The cluster head manages the nodes in the cluster, collects data collected by the members, and establishes a TDMA timing table for the member nodes. Then, send the timing table to the nodes in the cluster. All nodes send the collected data to the cluster head according to the time slot specified in the timetable. The cluster head performs simple preprocessing on the data in the cluster and then sends it to the upper node. At this point, one “round” is over and the next cycle begins.

The article "Smart Garden Planning and Design Based on the Agricultural Internet of Things" was published in 2022. Journal: Comput Intell Neurosci.

Although the LEACH protocol has a very good performance in long-term monitoring, it also has some shortcomings, mainly including the following aspects:

1. In each round of cluster establishment, all nodes must participate, and the amount of calculation is very large, which is a great waste of resources
2. The selection of the cluster head is random
3. All cluster capitals communicate directly with sink nodes and do not consider the resource loss caused by long-distance communication between cluster heads far away from sink nodes

This paper introduces a new meta-inspired optimization algorithm—gray wolf algorithm—to solve the above-mentioned problems of LEACH algorithm, so that it can better serve agricultural applications. Meta-heuristic algorithms are favored by researchers because of their simplicity and flexibility. The gray wolf (GWO) algorithm is currently the most popular meta-heuristic algorithm in theoretical research. The main idea of the algorithm is to simulate the social hierarchy and group hunting behavior of the gray wolf family in nature. Gray wolves belong to the canine family and like to live in groups. On average, each group consists of 5–12 gray wolves and follows a strict hierarchy, as shown in Figure 3.

The social status of wolves in the gray wolf family can be divided into 4 levels from top to bottom, namely, *α* wolves, *β* wolves, *δ* wolves, and *ω* wolves. Alpha wolf is a wolf, mainly responsible for deciding the time and place of sleeping, hunting, and tactics. The second level of the gray wolf class is *β* wolves. *β* wolves are subordinate wolves, mainly responsible for assisting the wolves to manage the wolf pack. When the wolf pack lacks alpha wolves, beta wolves will replace alpha wolves. The delta wolf is on the third level. The delta wolf obeys the instructions of the alpha wolf and the beta wolf, but it can command the *ω* wolf at the bottom. The *ω* wolf is mainly responsible for balancing the relationships within the population.

The collective hunting of gray wolves is an important part of the social activities of gray wolves. Scholars such as Muro have introduced the hunting behavior of gray wolves in detail in the literature, as shown in Figure 4.

Mathematical model of gray wolf algorithm: (1) to establish a mathematical model of gray wolf's social hierarchy, we named the solution with the best fitness as *α* wolf. Therefore, the second and third best solutions are named *β* wolves as well as *ω* wolves, respectively.

The article "Smart Garden Planning and Design Based on the Agricultural Internet of Things" was published in 2022. Journal: Comput Intell Neurosci.

### 3.1. Hunting Model

In order to simulate the encircling behavior of gray wolves with a mathematical model, equations (6) and (7) are introduced.

(6) $$\begin{array}{c} \overset{⟶}{D}=\left|\overset{⟶}{C}\overset{⟶}{X_{P}}\left(t\right)-\overset{⟶}{X}\left(t\right)\right|, \end{array}$$

(7) $$\begin{array}{c} \overset{⟶}{X}\left(t+l\right)=\overset{⟶}{X_{p}}\left(t\right)-\overset{⟶}{A}\overset{⟶}{D}. \end{array}$$

The calculation formulas for vectors $\overset{⟶}{A}$ and $\overset{⟶}{C}$ are as follows [22]:

(8) $$\begin{array}{c} \overset{⟶}{A}=2\overset{⟶}{a}\overset{⟶}{r_{1}}-\overset{⟶}{a},\\ \overset{⟶}{C}=2\overset{⟶}{r_{2}}. \end{array}$$

### 3.2. Attack Model

GWO hunts are led by *α*, and *β* and 8 occasionally participate. In order to mathematically simulate the hunting behavior of gray wolves, we assume that *α* (the best candidate solution) and *β* and 6 have a more accurate understanding of the potential location of the prey. Therefore, the algorithm saves the first three optimal solutions obtained so far and forces other search agents (include o) to update their positions according to the position of the best search agent. And its update formula is as follows:

(9) $$\begin{array}{c} \overset{⟶}{D_{\alpha }}=\left|\overset{⟶}{C_{1}}\overset{⟶}{X_{\alpha }}-\overset{⟶}{X}\right|, \end{array}$$

(10) $$\begin{array}{c} \overset{⟶}{D_{\beta }}=\left|\overset{⟶}{C_{2}}\overset{⟶}{X_{\beta }}-\overset{⟶}{X}\right|, \end{array}$$

(11) $$\begin{array}{c} \overset{⟶}{D_{\delta }}=\left|\overset{⟶}{C_{3}}\overset{⟶}{X_{\delta }}-\overset{⟶}{X}\right|, \end{array}$$

(12) $$\begin{array}{c} \overset{⟶}{X_{1}}=\overset{⟶}{X_{\alpha }}-\overset{⟶}{A_{1}}\left(\overset{⟶}{D_{\alpha }}\right), \end{array}$$

(13) $$\begin{array}{c} \overset{⟶}{X_{2}}=\overset{⟶}{X_{\beta }}-\overset{⟶}{A_{2}}\left(\overset{⟶}{D_{\beta }}\right), \end{array}$$

(14) $$\begin{array}{c} \overset{⟶}{X_{3}}=\overset{⟶}{X_{\delta }}-\overset{⟶}{A_{3}}\left(\overset{⟶}{D_{\delta }}\right), \end{array}$$

(15) $$\begin{array}{c} \overset{⟶}{X}\left(t+l\right)=\frac{\overset{⟶}{X_{1}}+\overset{⟶}{X_{2}}+\overset{⟶}{X_{3}}}{3}. \end{array}$$

Equations (12) to (14) define the length and direction of the advancement of *ω* wolf toward *α*, *β*, and *δ*, respectively. Equation (15) represents the current *α* position. And the specific process is shown in Figure 5.

The general steps of the GWO algorithm are as follows:

  Step 1: the algorithm initializes the wolf pack
  Step 2: the algorithm calculates the fitness value of each wolf
  Step 3: the algorithm selects the top three wolves with the best fitness as *α*, *β*, and 8
  Step 4: the algorithm uses formulas (9) to (14) to update other wolves (*ω*)
  Step 5: the algorithm updates parameters, a, A, and C
  Step 6: if the end condition is not met, the algorithm goes to step 2
  Step 7: the algorithm outputs the position of *α*

In this paper, sensor nodes represent individual wolves, and base station BS represents prey.

The article "Smart Garden Planning and Design Based on the Agricultural Internet of Things" was published in 2022. Journal: Comput Intell Neurosci.

HCGW adopts a round-robin mechanism similar to LEACH, and each round performs the following steps: ①According to the relationship between signal reception and transmission and distance, the simulated gray wolf algorithm divides the network into multiple layers. Each node determines which layer it is in based on the distance between its position and the base station. ②The fitness function includes the remaining energy of the node. ③After the cluster head is determined, all member nodes choose the cluster head to form a cluster. ④ The GWO communication route is established between the cluster heads to avoid long-distance transmission. ⑤Establishes a new route for route maintenance.

#### 3.2.1. Network Layering

As shown in Figure 6, this paper assumes that the network can be divided into *L* layers. According to energy model formulas (2)–(4), nodes with a distance less than *d*_0_ from the base station are classified as the first layer, and they are marked as layer *α* according to their priority. And the rest are *β* layer and 6 layer in order.

The node *SN*_*i*_ is in the lth layer:

(16) $$\begin{array}{c} l=\left[2\times \frac{d_{i}}{d_{0}}\right]. \end{array}$$

By layering the nodes, the communication distance between cluster heads is less than or equal to *d*_0_ during data transmission, which can effectively avoid the energy loss caused by long-distance communication.

#### 3.2.2. Cluster Head Selection Method Based on Fitness Principle

After the sensor nodes are layered, in each layer, the fitness function and fitness rules are used to calculate the fitness of the node, and one or several nodes with high fitness are selected as the cluster head of this layer.

*(1) Node Remaining Energy*. The node's remaining energy *E*_RE_ represents the maximum energy left by the node after a number of rounds in the network.

(17) $$\begin{array}{c} E_{\text{RE}}=E_{\text{init}}-E_{r}. \end{array}$$

*(2) Node Density*. The greater the node density, the more neighbor nodes of the node, and the less energy it consumes when exchanging data with surrounding nodes. The node density is represented by *P*_*SN*_*i*__, and its calculation company is as follows:

(18) $$\begin{array}{c} P_{SN_{i}}=\frac{N}{\pi \cdot d_{0}^{2}}. \end{array}$$

Here, N is the number of nodes in the communication range of *d*_0_.

*(3) Node Centrality C*. The centrality C represents the average distance between a certain node SN and its neighboring nodes. The smaller C is, the closer it is, the less energy is needed for communication, and vice versa.

(19) $$\begin{array}{c} C_{i}=\sqrt{{\left(x_{i}-\frac{1}{n}\sum_{j}^{n}x_{j}\right)}^{2}+{\left(y_{i}-\frac{1}{n}\sum_{j}^{n}y_{j}\right)}^{2}}. \end{array}$$

Here, *x*_*i*_ represents the abscissa of node *SN*_*i*_, and *y*_*i*_ represents the ordinate of node *SN*_*i*_.

*(4) Fitness Function*. The cluster head selection is determined by the fitness function. In the GWO algorithm, the fitness function plays a very important role in finding the prey mechanism. The input of this function is the characteristics of the node, including node residual energy (*E*_RE_), node density, and node centrality. And, the output is the fitness value of whether the node can become the cluster head.

(20) $$\begin{array}{c} f\left(CH_{i}\right)=q_{1}\left|\frac{P_{SN_{i}}}{C_{i}}\right|+q_{2}\sum E_{\text{RE}}. \end{array}$$

Here, *q*_1_ and *q*_2_ are random numbers in the range of [0, 1]. A certain threshold is set for the fitness, and the node with a fitness value greater than this threshold will be selected as the cluster head.

*(5) Fitness Rules*. The HCGW algorithm uses adaptive criteria for comprehensive evaluation. The nodes with more residual energy, higher node density, and higher centrality have very high priority. HCGW contains a total of 3 3*∗*3*∗*=27 fitness criteria, as shown in Table 1.

The article "Smart Garden Planning and Design Based on the Agricultural Internet of Things" was published in 2022. Journal: Comput Intell Neurosci.

#### 3.2.3. Formation of the Family

After receiving the Invite.Msg message, the member node calculates the approximate distance *d* from itself to each CH and selects the cluster head with the smallest distance to join to form a cluster structure.

#### 3.2.4. Route Establishment and Maintenance

The cluster head performs preprocessing steps such as compression and optimization of the data. Then, the algorithm sends the data head node of the upper layer with higher priority according to the priority order of the hierarchy and then transmits it in turn until the first layer. At this time, a multihop routing similar to the gray wolf hierarchy is established.

After a long enough time *T*, the routing of the entire network will be updated. Compared with the LEACH protocol's global mechanism, proposed by the HCGW algorithm, it can greatly save computational and broadcast costs and at the same time achieve local optimality.

## 4. Smart Garden Planning and Design Based on the Agricultural Internet of Things

The process for the smart garden information management platform to access and call basic geographic data is as follows: (1) The smart garden information management platform sends a graphical call request to the basic geographic information sharing service platform. (2) After receiving the graphic data query request, the basic geographic information sharing service platform will execute the relevant graphic data query process, package the query results (map images or JSON format attribute data), and return them to the smart garden information management platform. (3) After receiving the query result, the intelligent garden information management platform displays it in the map window of the platform. The thematic geographic data of landscaping is directly accessed and invoked on the platform and can be displayed superimposed with the basic geographic information sharing service. The schematic diagram of the business data interface model (process) of the smart garden information management platform is shown in Figure 7.

The article "Smart Garden Planning and Design Based on the Agricultural Internet of Things" was published in 2022. Journal: Comput Intell Neurosci.

After constructing a smart garden planning system based on the agricultural Internet of Things, the effect of the data processing of the agricultural Internet of Things in this paper is evaluated, and a garden simulation system is constructed to analyze the performance of the system. The network nodes of the simulation system are shown in Figure 8.

Through the performance verification of the above model, the data processing effect of the agricultural smart garden is shown in Table 2 and Figure 9.

The above model verifies the data processing effect of the agricultural smart garden system.

On this basis, the planning and design effects of agricultural smart gardens are carried out, and the results shown in Table 3 and Figure 10 are obtained.

The above analysis verifies that the smart garden planning and design system has a good planning and design effect.

## 5. Conclusion

People can intuitively watch the objects in the real environment scene through the network platform and can select corresponding operations on the network client to perform corresponding operations on the real objects in the real environment. Virtual experience is dependent on computer and Internet of Things technology. Compared with real experience, virtual experience has some inherent characteristics, such as virtual experience, virtual experience with uncertainty, and virtual experience with globality. This paper combines the agricultural Internet of Things technology to carry out smart garden planning and design. With the theme of agricultural pastoral, it promotes industrial development and raises people's awareness of ecological and environmental protection and brings people a good pastoral scenery experience.

The article "Smart Garden Planning and Design Based on the Agricultural Internet of Things" was published in 2022. Journal: Comput Intell Neurosci.

## Figures and Tables

**Figure 1:** Schematic diagram of LEACH protocol clustering.

**Figure 2:** LEACH protocol flowchart.

**Figure 3:** Schematic diagram of the gray wolf population hierarchy.

**Figure 4:** Gray wolf hunting behavior. (a) Chasing, approaching, and tracking prey. (b) Pursuit, harassment, and encirclement. (c) Static state and attack.

**Figure 5:** Schematic diagram of the gray wolf algorithm.

**Figure 6:** Schematic diagram of network layering.

**Figure 7:** Schematic diagram of the data interface model of the smart garden business.

**Figure 8:** Model of the agricultural smart garden system.

**Figure 9:** Data processing statistics.

**Figure 10:** Statistical diagram of planning and design effects of smart gardens.

**Table 1:** Fitness rules.

Fitness rules	Remaining energy	Node density	Centrality	Adaptability
1	Few	Secondary	Secondary	Very secondary
2	Few	Secondary	Commonly	Very secondary
3	Few	Secondary	High	Very secondary
4	Few	Commonly	Secondary	Very secondary
5	Few	Commonly	Commonly	Very secondary
6	Few	Commonly	High	Very secondary
7	Few	High	Secondary	Very secondary
8	Few	High	Commonly	Very secondary
9	Few	High	High	Very secondary
10	Commonly	Secondary	Secondary	Slightly secondaryer
11	Commonly	Secondary	Commonly	Slightly secondaryer
12	Commonly	Secondary	High	Commonly
13	Commonly	Commonly	Secondary	Slightly secondaryer
14	Commonly	Commonly	Commonly	Commonly
15	Commonly	Commonly	High	Slightly higher
16	Commonly	High	Secondary	Slightly secondaryer
17	Commonly	High	Commonly	Commonly
18	Commonly	High	High	Slightly higher
19	Many	Secondary	Secondary	Slightly secondaryer
20	Many	Secondary	Commonly	Commonly
21	Many	Secondary	High	Slightly higher
22	Many	Commonly	Secondary	Commonly
23	Many	Commonly	Commonly	Slightly higher
24	Many	Commonly	High	High
25	Many	High	Secondary	Commonly
26	Many	High	Commonly	High
27	Many	High	High	Very high

**Table 2:** Data processing effect of agricultural IoT smart garden.

No.	Data processing	No.	Data processing	No.	Data processing
1	95.29	16	93.11	31	93.52
2	92.29	17	96.08	32	93.08
3	93.11	18	94.79	33	96.04
4	96.55	19	92.66	34	96.12
5	93.31	20	93.90	35	93.71
6	95.61	21	95.89	36	96.00
7	93.67	22	93.83	37	93.68
8	96.33	23	93.08	38	92.51
9	94.56	24	94.35	39	94.51
10	94.57	25	93.43	40	95.17
11	94.10	26	95.76	41	93.12
12	93.86	27	95.91	42	92.83
13	94.01	28	92.62	43	94.63
14	95.69	29	94.79	44	95.69
15	92.56	30	94.09	45	95.47

**Table 3:** Planning and design effects of agricultural smart gardens.

No.	Planning and design	No.	Planning and design	No.	Planning and design
1	86.45	16	82.77	31	81.62
2	74.26	17	80.81	32	89.68
3	80.49	18	88.72	33	77.24
4	89.06	19	86.27	34	88.22
5	82.10	20	80.38	35	83.12
6	84.06	21	86.88	36	74.41
7	85.45	22	74.03	37	80.85
8	89.51	23	82.76	38	91.39
9	74.47	24	74.25	39	78.90
10	86.67	25	80.52	40	79.56
11	83.42	26	80.94	41	74.14
12	78.27	27	82.41	42	90.94
13	73.73	28	85.22	43	87.79
14	88.74	29	84.31	44	81.33
15	77.87	30	82.94	45	88.75

The article "Smart Garden Planning and Design Based on the Agricultural Internet of Things" was published in 2022. Journal: Comput Intell Neurosci.

## Data Availability

The data used to support the findings of this study are available from the corresponding author upon request.
